# Data Analysis and Computational Methods for Assessing Knowledge of Obesity Risk Factors among Saudi Citizens

**DOI:** 10.1155/2021/1371336

**Published:** 2021-10-26

**Authors:** Alanazi Talal Abdulrahman, Dalia Kamal Alnagar

**Affiliations:** ^1^Department of Mathematics, University of Ha'il, Saudi Arabia; ^2^Department of Statistics, University of Tabuk, Saudi Arabia; ^3^Department of Statistics, Omdurman Islamic University, Sudan

## Abstract

**Introduction:**

According to the World Health Organization (2020), obesity is a growing problem worldwide. In fact, obesity is characterized as an epidemic.

**Objective:**

The aim of this paper is to use a logistic regression model as one of the generalized linear models and decision tree as one of the machine learning in order to assess the knowledge of the risk factors for obesity among citizens in Saudi Arabia.

**Methods and Materials:**

A cross-sectional questionnaire was given to the general population in KSA, using Google forms, to collect data. A total of 1369 people responded.

**Results:**

The findings showed that there is widespread knowledge of risk factors for obesity among citizens in Saudi Arabia. Participants' knowledge of risk factors was very high (95.5%). In addition, a significant association was found between demographics (gender, age, and level of education) and knowledge of risk factors for obesity, in assessing variables for knowledge of the risk factors for obesity in relation to the demographics of gender and level of education. In addition, from decision tree results, we found that level of education and marital status were the most important variables to affect knowledge of risk factors for obesity among respondents. The accuracy of correctly classified cases was 95.5%, the same in logistic regression and decision tree.

**Conclusion:**

The majority of participants saw regular exercise and diet as an essential way to reduce obesity; however, awareness campaigns should be maintained in order to avoid complacency and combat the disease.

## 1. Introduction

According to the World Health Organization, obesity is a growing problem worldwide. In fact, obesity is characterized as an epidemic, affecting nearly 650 million adults worldwide. Specifically, about 13% of the adult population worldwide is considered obese [1].

In Saudi Arabia, obesity is a growing problem. A systematic analysis of data from 33 years before 2014 revealed that Saudi Arabia was one of the top seven countries with the most severe rises in both male and female obesity rates [2]. Nearly 35% of Saudi adults are obese, with females having higher rates than males (41% vs. 31%) [3]. There was evidence to suggest that obesity is set to worsen in the decades to come [4]. Obese persons are more likely to develop heart disease, hypertension, stroke, type 2 diabetes, and other adverse health outcomes than nonobese persons. From an economic perspective, obesity costs the country about $147 billion in 2008 American dollars annually, and the annual cost is rising substantially over the past 10 years or so.

A variety of studies addressed the topic of obesity and its causes, which provided statistical data that show its prevalence and the associated factors. Among these studies is a study by Mosli et al. [5], which discovered the association between educational level and income level with odds of being obese among adults in KSA. In contrast to participants with advanced education or higher, ignorant participants and those with rudimentary schooling had higher chances of corpulence. In any case, members with low pay had lower chances than members who had higher pay.

A study by Al-Raddadi et al. [6] is aimed at studying the relationship of demographic and way of life factors, recently demonstrated to be related to overabundant weight in different populaces, and BMI in the grown-up populace of Jeddah of KSA. In the study, there were 1419 persons: 667 males and 752 females. 30.1% males and 35.6% females were the prevalence of overweight and obesity, the prevalence increased to 60 years, and it decreased in the older age group in both genders. In males, the risk of obesity increased with obtaining a postgraduate degree, and the rate decreases with increased physical activity, and in females, obesity increased the risk of prediabetes and diabetes; the risk of prediabetes, diabetes, dyslipidemia, and hypertension increases with increasing BMI.

The study of Al-Qahtani [7] was aimed at appraising the commonness of overweight and obesity among grown-ups going to essential medical service settings, southwestern district of the KSA. Data on BMI estimation was recorded for 1649 out of 1681 individuals (98.1%). The general mean weight was 74.1 ± 15.81 kg, and that for males was 77.69 ± 16.14 kg versus 69.37 ± 14.02 kg for females. The general predominance of overweight and stoutness was, individually, 38.3% and 27.6%. Smoking was not essentially connected with corpulence, though hypertension was altogether connected with weight. The danger of overweight or corpulence essentially expanded from the most elevated to the least month-to-month pay. High spread of obesity and overweight should be considered a public health worry to be trailed by explicit mediations at the network level with multidisciplinary exercises beginning from childhood as an early stage counteraction program.

The point of the study of Aljabri et al. [8] was to assess obesity and overweight in Saudi women of childbearing age. Age was 32.3 ± 9.1 years (least 15 and most extreme 49 years), 5.8% (165) were lean, 26.6% (759) were of typical weight, 27.6% (785) were overweight, 22.4% (637) were obese Grade I, and 11.1% (316) were large Grade II while 6.6% (187) were beefy beyond belief (obese Grade III). The recurrence of overweight and stoutness expanded with the advance of age gathering, and dismal corpulence was most elevated in the 40-long-term age gathering. Except if quick advances are taken to contain the expanding commonness of weight, the medical care costs for ongoing sicknesses will represent a colossal budgetary weight to the KSA.

Albin Saleh et al. [9] assessed obesity commonness among kids and teenagers in Al-Ahsa, KSA, for the year 2016 and decided the connected preventable danger factors. Obesity and overweight were 29.6% (10.8% overweight, 3.8% fat, and 15% obese large). The prevalence of obesity and overweight was altogether connected with youth weight, parental overweight, mother's work, family pay, fast food, actual dormancy, and time spent sitting in front of the TV. There is an earnest need to spread mindfulness about obesity, and the anticipation programs that include schools and families are the vital systems for controlling the current epidemic of overweight and obesity.

Alshammari and Elasbali [10] measured the prevalence paces of obesity in Hail City in KSA. 80.83% (1455/1800) have fully responded to all required parameters of the 1800, 52% (756/1455) were females and 48% (699/1455) were males, and 60.34% (878/1455) were found obese and overweight, with females' proportion more than males. Obesity and overweight are common in Hail City in KSA with generally higher females' susceptibility.

Al-Hazzaa et al. [11] sought to give updated estimates of obesity and overweight prevalence from three main cities in Saudi Arabia, namely, Riyadh, Al-Khobar, and Jeddah, with members of 2,908 auxiliary school understudies aged 14 to 19 years; the prevalence of overweight was 19.5 percent in individuals and 20.8 percent in girls, while stoutness was 24.1 percent in males and 14 percent in females. The predominance of obesity in males and females was 35.9% and 30.3%, respectively. Such high pervasiveness of obesity and overweight is a significant public health concern.

Al-Ateeq and Al-Hargan [12] looked at the potential relationship between obesity and the method of transportation to neighborhood offices, social climate, type of work, and actual movement at neighborhood offices and at home. Of the participants, 33.7% were overweight and only 39.2% were obese. Most of the members traveled to work (98%), school (90.2%), shopping centers (95.7%), eateries (91.5%), social visits (84%), mosques (84.3%), and markets (50.2%). The rate of obesity was higher among members who drove (45%) than among those who walked (30%) to the market stores. Thus, the proposed paper's principal goal is to assess the knowledge of the risk factors for obesity among citizens in Saudi Arabia towards the risk factors for obesity.

Knowledge is the ability to learn, retain, and apply knowledge; it is a combination of comprehension, experience, discernment, and skill.

Many researches have reported the varied prevalence of obesity and overweight among Saudi residents, but there is little information on individuals' knowledge of the risk factors for obesity. As a result, the findings of this study are critical since they will assist in the management of obesity.

Nonetheless, there has been an expanded interest in defining new factual models or new groups of measurable models to give a superior depiction of the issues viable. For more details, we refer to Abdulrahman and Alamri [13] and Abdulrahman [14].

## 2. Materials and Methods

### 2.1. The Questionnaire

A questionnaire was used in this assessment to allow individuals to identify obesity risk factors. The questionnaire comprised two sections. Section one included questions on personal information, including gender, age, marital status, educational qualifications, and occupation. The other section contained ten questions on the causes of obesity. The participants were asked to determine the main cause of obesity among the following reasons:

- Heredity is one of the most important causes of obesity
- Diet pattern has a significant impact on the causes of obesity
- Consumption of sugars and starches is a major cause of obesity
- Lack of exercise is a major cause of obesity
- Lack of sleep of a person may expose him to obesity
- Some hormones such as leptin can increase obesity
- Taking some medications may expose a person to obesity
- As a person gets older, he is at risk of obesity
- Some diseases that affect a person are exposed to obesity
- Mental state is one of the most important causes of obesity

The target populace was 748 male responders and 621 female respondents.

### 2.2. Data Analysis and Study Test

Table 1 shows demographic characteristics such as age, gender, education level, marital status, and work. All participants spoke Arabic fluently. SPSS version 25.0 was used to analyze the data. Quantitative analysis entailed calculating frequencies and percentages for demographic data, which were then tested using inferential statistics. Pearson's chi-squared test was used to evaluate the analyses' goodness of fit; homogeneity, to compare respondents (groups) in a specified variable; and independence, to determine whether respondent cohorts exhibited distinct answers.

### 2.3. Binary Logistic Regression Model

Binary logistic regression is a statistical method used to investigate a variety of subjects in medical research [15, 16]. It helps researchers to predict whether an event will occur or not based on predictor factors [17].

The odds ratios for each of the model's independent variables (age, gender, marital status, level of education, and work) were estimated using logistic regression. When the odds ratio is more than one, it shows a positive relationship, and when it is less than one, it suggests a negative correlation. To forecast a logit transformation of the likelihood of the presence of the attribute of interest, use the following formula:

(1) $$\begin{array}{c} \text{Logit}\left(p\right)=b_{0}+b_{1}X_{1}+b_{2}X_{2}+\cdots +b_{k}X_{k}. \end{array}$$

Here, *p* is the probability of the occurrence of the property of interest.

The logged chances are defined as the logit transformation:

(2) $$\begin{array}{c} \text{Odds}=\frac{p}{1-p}. \end{array}$$

Here, *p* indicates the probability of a characteristic's presence, 1 − *p* represents the probability of a characteristic's absence, and

(3) $$\begin{array}{c} \text{Logit}\left(\text{p}\right)=\text{loglog}\frac{p}{1-p}. \end{array}$$

The logit is a function that translates probability values from (0, 1)(0, 1) to real numbers (−∞, ∞).

### 2.4. Decision Tree

A decision is a flowchart-like structure in which each internal node represents a test on an attribute, each branch of the tree represents a test outcome, and each leaf node stores a class label.

The Chi-square Automatic Interaction Detector (CHAID) method utilized in this research detects such differences by employing two tests to assess the relationship between the dependent and independent variables [18]. The CHAID process begins by identifying independent variables that have a statistically significant relationship with the dependent or target variable.

Decision tree techniques may be used to choose the most relevant input variables that should be utilized to build decision tree models, which can then be used to formulate clinical hypotheses and inform further research.

The data mining technique of decision tree analysis offers an alternative means of identifying specific variables affected by knowledge of the risk factors for obesity among the respondents, which included the model of participants' gender, age, marital status, education, level of education, and work.

The information gain may be used to select the appropriate attribute to utilize for data classification:

(4) $$\begin{array}{c} G\left(A\right)=I\left(p,n\right)-\overset{v}{\underset{i=1}{\sum }}\frac{p_{i+n_{i}}}{p+n}I\left(p_{i},n_{i}\right), \end{array}$$

where *p* is the probability that the tuple belongs to class V and *n* is the number of attributes in the class:

(5) $$\begin{array}{c} I\left(p,n\right)=\frac{p}{p+n}\log_{2}\frac{p}{p+n}-\frac{p}{p+n}\log_{2}\frac{n}{p+n\;}. \end{array}$$

A binary outcome value for the *i* object is represented by *n* and *p* and takes zero and one values [17].

## 3. Results

The reliability analysis result showed that Cronbach's alpha was 0.68 for 10 items. Therefore, there was internal consistency of the scales. Hence, this instrument used in this study had a high reliability value (Alnagar et al. [19]).

The demographic information is shown in Table 1. Of the 1369 samples analyzed, *n* = 748 (54.6%) were male and *n* = 621 (45.4%) were female; the majority of the participants' (*n* = 602, 44.0%) ages range from 18 to30 while the percentage of respondents with ages less than 18 was *n* = 76 (5.6%).

According to their marital status, *n* = 871 (63.6%) of respondents are married and *n* = 498 (36.4%) are unmarried. The majority of participates were university students (*n* = 923, 67.4%) while the percentage of respondents with postgraduate education levels were *n* = 186 (13.6%).

Table 2 shows that the participants' knowledge of the risk factors for obesity was very high (95.5%). Specifically, they were most knowledgeable about diet (99.3%), fast food (96.6%), heredity (74.3%), lack of exercise (93.5%), lack of sleep (82.8%), hormones (98.2%), increased age (67.3%), some diseases (90.4%), and mental stress (87.1%).

Table 3 shows the association between several demographic variables and knowledge of risk factors for obesity among respondents; females had significantly higher (97.1%) knowledge of risk factors for obesity than males (94.3%). Moreover, respondents of age ranging from 30 to 40 had significantly higher (96.7%) knowledge of risk factors for obesity than those of ages less than 18 (88.2%). Majority of the respondents married had 96.1% high knowledge of risk factors for obesity than those unmarried (94.9%), so there was no association between knowledge of risk factors for obesity and marital status.

University students had significantly higher (96.9%) knowledge of risk factors for obesity than primary and middle school students (94.3%). Private workers had high (96.6%) knowledge of risk factors for obesity than those that do not work (95.1%), so there is no association between knowledge of risk factors for obesity and work.

In sum, there were associations between knowledge of risk factors for obesity among the respondents and variables (gender, age, and level of education).

Table 4 shows a binary logistic regression model to estimate variables affected on knowledge of risk factors for obesity among respondents, including the model of participants' gender, age, marital status, education, level of education, and work. Items emerged as significant (*p* ≤ 0.05) from the logistic regression analysis model; we found that gender and level of education were both variables affecting knowledge of risk factors for obesity among respondents. Gender as a variable showed a good odds ratio of 2.261 at 95% confidence interval (CI = 1.189, 4.301). There was a high knowledge of risk factors for obesity among respondents from those with level of education, with odds ratio = 2.054 (95% CI = 1.426, 2.957).

The classification results for the decision tree for knowledge of risk factors for obesity among respondents are shown in Table 5. The percentages of cases that were correctly classified were 95.5%, which demonstrates the accuracy of the decision tree model.

Table 6 shows that decision trees were used to gain information to determine which variables are most important to affect knowledge of risk factors for obesity among respondents. Age, level of education, and marital status were the most important variables to affect knowledge of risk factors for obesity among respondents.

## 4. Discussion and Conclusion

The findings of this study are that there is widespread knowledge of risk factors for obesity among citizens in Saudi Arabia; it agrees with [20]. The participants' knowledge of obesity risk factors was generally high (95.5%). In addition, there was a high knowledge of risk factors for obesity among respondents from those with a level of education. A significant association was found between demographics (gender, age, and level of education) and knowledge of risk factors for obesity; it agrees with [21]. A decision tree was used to gain information to determine which variables are most important to affect knowledge of risk factors for obesity among respondents; the percentages of cases that were correctly classified are 95.5%, which demonstrates the accuracy of the decision tree model.

Accuracy of correctly classified cases was the same in two methods. However, the results are different in the logistic regression and decision tree; in the logistic regression analysis model, we found that both gender and level of education variables affected knowledge of risk factors for obesity among respondents. Age, level of education, and marital status were the most important variables to affect knowledge of risk factors for obesity among respondents.

Logistic regression is a statistical approach for modeling the probability *p* of an occurrence in terms of one or more predictor variables' values. The model is made up of two parts: a binary tree structure that depicts the data divisions and a series of basic linear logistic models, one for each partition. This is the division of model complexity that makes the model easy to interpret. In conclusion, the majority of participants saw regular exercise and diet as an essential way to reduce obesity; however, awareness campaigns should be maintained in order to avoid complacency and combat the disease.

## Figures and Tables

**Table 1:** The demographic information.

Variable	Frequency	Percent
Gender		
Male	748	54.6
Female	621	45.4
Age		
Less than 18	76	5.6
18-30	602	44.0
30-40	394	28.8
40 and more	297	21.7
Marital status		
Married	871	63.6
Unmarried	498	36.4
Level of education		
Primary and middle school	45	3.3
Secondary school	215	15.7
University student	923	67.4
Postgraduate	186	13.6
Work		
Government employee	616	45.0
Private sector	177	12.9
I do not work	576	42.1

**Table 2:** Participants' knowledge of the risk factors for obesity.

Variable	Knowledge	Percent
Poor knowledge	61	4.5
Good knowledge	1308	95.5
Heredity	1018	74.3
Diet	1359	99.3
Fast food	1322	96.6
Lack of exercise	1280	93.5
Lack of sleep	1134	82.8
Some hormones	1344	98.2
Taking some medications	1300	95
The older a person	930	67.9
Some diseases	1238	90.4
Mental stress	1192	87.1

**Table 3:** Association between several demographic variables and knowledge of risk factors for obesity among respondents.

Variable	Poor	Good	*p* value
Gender			0.001
Male	43 (5.7%)	705 (94.3%)	
Female	18 (2.9%)	603 (97.1%)	
Age			0.007
Less than 18	9 (11.8%)	67 (88.2)	
18-30	29 (4.8%)	573 (95.2%)	
30-40	13 (3.3%)	381 (96.7%)	
40 and more	10 (3.4%)	287 (96.6%)	
Marital status			0.191
Married	34 (3.9%)	837 (96.1%)	
Unmarried	27 (5.4%)	471 (94.6)	
Level of education			0.001
Primary and middle school	8 (17.8%)	37 (82.2%)	
Secondary school	18 (8.4%)	197 (91.2%)	
University student	29 (3.1%)	894 (96.9%)	
Postgraduate	6 (3.2%)	180 (96.8%)	
Work			0.704
Government employee	27 (4.4%)	589 (95.6%)	
Private work	6 (3.4%)	171 (96.6%)	
I do not work	28 (4.9%)	548 (95.1%)	

**Table 4:** Binary logistic regression model to estimate variables affecting knowledge of risk factors for obesity among respondents.

Variable	Standard error	*p* value	Odds ratio	95% CI for odds ratio	
				Lower	Upper
Age	0.189	0.061	1.424	0.983	2.063
Gender	0.328	0.013	2.261	1.189	4.301
Marital status	0.354	0.748	1.121	0.560	2.242
Level of education	0.186	0.001	2.054	1.426	2.957
Work	0.182	0.845	0.965	0.675	1.379
Constant	1.062	0.335	0.359		

**Table 5:** Classification table for the decision tree for knowledge of risk factors for obesity among respondents.

Observed	Predicted	Observed	Predicted
Poor knowledge	0	61	0.0%
Good knowledge	0	1308	100.0%
Overall percentage	0.0%	100.0%	95.5%

Growing method: Classification Regression Tree (CRT). Dependent variable: knowledge.

**Table 6:** Variable importance using CART methods.

Independent variable	Importance	Normalized importance
Age	0.002	100.0%
Level of education	0.002	90.7%
Marital status	0.001	35.5%
Work	0.000	22.0%
Gender	0.000	11.7%

Growing method: CRT. Dependent variable: knowledge.

## Data Availability

The data that support the findings of this study are available on request from the corresponding author.
